# Effect of Apatinib Combined with Seggio on the Expression of Serum AFP and CA724 and Long-Term Survival Rate in Patients with Advanced Gastric Cancer Undergoing Comfortable Nursing Intervention

**DOI:** 10.1155/2022/2004973

**Published:** 2022-04-07

**Authors:** Dawei Ren, Mi Feng, Shengmin Zhang, Yun Zhang, Ji Li

**Affiliations:** ^1^Department of General Surgery, Qilu Hospital (Qingdao), Cheeloo College of Medicine, Shandong University, Qingdao 266035, Shandong, China; ^2^Department of General Surgery, Jiakang Hospital, Jiakang 276000, China; ^3^PIVAS, The Affiliated Qingdao Central Hospital of Qingdao University, The Second Affiliated Hospital of Medical College of Qingdao University, Qingdao 266042, Shandong, China; ^4^Department of Pediatrics, Zhangqiu District People's Hospital, Jinan 250200, China; ^5^Department of Pharmacy, Qilu Hospital (Qingdao), Cheeloo College of Medicine, Shandong University, Qingdao 266035, Shandong, China

## Abstract

**Objective:**

To study the effect of apatinib combined with seggio on the expression of serum AFP and CA724 and the long-term survival rate in advanced gastric cancer patients undergoing comfort nursing intervention.

**Methods:**

98 advanced gastric cancer patients were divided into single-drug group and joint group. Both groups of patients were given comfort nursing intervention, the single-drug group was treated with seggio, and the joint group was treated with apatinib and seggio. The clinical efficacy, survival rate, relationship between the tumor markers and the survival time, serum tumor markers levels (CA724 and AFP), inflammatory factors (IL-4, IL-10) levels, quality-of-life scores, and immunity function were measured after treatment.

**Results:**

The clinical efficacy in the joint group was better than that in the single-drug group. The three-year survival time in the joint group was upregulated relative to the single-drug group. The patients with high expression of CA724 or AFP had a lower survival time than the patients with low expression of CA724 or AFP. After treatment, IL-10 and IL-4 levels were obviously decreased, and the joint group showed a more obvious decrease compared with the single-drug group. The quality-of-life scores were significantly upregulated after treatment, and compared with the joint group, the scores in the single drug-group were obviously higher. The CD4+/CD8+, CD4+, and CD3+ levels were increased, while CD8+ levels were decreased after treatment, and the changes of each index in the joint group were more significant than those in the single-drug group. The content of CA724 and AFP were significantly decreased after treatment, and the joint group showed a more significant decrease than the single-drug group.

**Conclusion:**

Apatinib combined with seggio for advanced gastric cancer patients' treatment based on comfort nursing intervention can improve the clinical efficacy and survival time, reduce inflammatory factors and serum tumor markers levels, enhance patients' immune function, and quality of life.

## 1. Introduction

Gastric cancer is a common digestive tract malignant tumor generated from gastric mucosal epithelial cells, which is related to improper diet, helicobacter pylori infection, genetic factors, etc. [1]. Its morbidity and mortality are high and increasing year by year, ranking the third among the related causes of death caused by malignant tumors worldwide [2]. China is a country with a high incidence of gastric cancer, and its mortality ranks second among malignant tumors in my country [3]. After endoscopic or surgical treatment of early gastric cancer, the 5-year survival rate can reach more than 90% [4]. However, the early symptoms of gastric cancer are often atypical. Most of the patients have reached the middle and late stages when they go to the doctor, who lose the opportunity for surgery. The 5-year survival rate is only about 20% [5], which seriously threatens the life safety of patients. Patients with advanced gastric cancer are difficult to be cured by surgery, and chemotherapy is needed to relieve clinical symptoms, control disease progression, and prolong survival.

Clinical studies have found that [6, 7], compared with traditional chemotherapy, molecular targeted therapy has obvious advantages, it can selectively kill tumor cells, and it is not easy to cause adverse reactions in patients, and the treatment safety is high, which has become the first choice for clinical treatment advanced gastric cancer patients in recent years. Judging from the clinical research results in the past 10 years, the wide application of molecular targeted therapy has greatly improved the prognosis of tumor diseases, especially in the treatment of colorectal cancer [8], lung cancer [9], and breast cancer [10]. Although the effect is very significant, the results achieved in the treatment of advanced gastric cancer are limited. Apatinib [11] is a targeted anticancer drug whose main mechanism of action is to block the downstream signal transduction of VEGF and VEGFR by acting on the ATP-binding site of VEGFR-2. It inhibits the formation of new blood vessels in tumors, makes the tumor lack of oxygen and nutrients during the process of tumor progression, and then stops development. It has good safety and can significantly prolong the survival of patients in combination with conventional chemotherapy. Gastric cancer patients mostly show pain and weight loss. This is mainly because gastric cancer patients generally have eating disorders, so they are prone to malnutrition, body weight continues to decline, and the patient's body resistance is reduced, which has great adverse effects on the treatment and rehabilitation of the disease. Comfortable nursing [12] belongs to a new type of nursing and is widely used in other clinical departments, mainly to provide patients with comprehensive and high-quality nursing services to ensure clinical efficacy.

In this study, we hypothesized that apatinib combined with seggio could improve the clinical efficacy and survival time of the patients with advanced gastric cancer. On the basis of high-quality nursing, apatinib combined with seggio was used to treat patients to observe the clinical efficacy and prognostic value of this method.

## 2. Materials and Methods

### 2.1. General Information

98 advanced gastric cancer patients were recruited from the above hospital from March 2016 to January 2018 and divided into joint group (*n* = 49) and single-drug group (*n* = 49). Single-drug group: 32 males and 17 females and age ranged from 42 to 71 years old, with an average age of (61.4 ± 13.7) years old. Tumor sites: 21 cases of gastric antrum, 12 cases of gastric body, and 16 cases of cardia. Clinical stage: 15 cases of stage IIIb, 23 cases of stage IIIc, and 11 cases of stage IV. There were 30 males and 19 females in the joint group, aged 45–73 years, with an average age of (62.6 ± 12.9) years old. Tumor sites: 23 cases of gastric antrum, 13 cases of gastric body, and 13 cases of cardia. Clinical stage: 12 cases of stage IIIb, 25 cases were in stage IIIc, and 12 cases were in stage IV. Inclusion criteria: (1) meeting the relevant diagnostic criteria for gastric cancer [13]; (2) confirmed by pathology or cytology and other laboratory tests; (3) clinical stage—IIIb to IV; (4) all patients signed an informed consent; and (5) the expected survival time of the patients was more than 6 months. Exclusion criteria: (1) complicated with organ failure; (2) associated with mental illness, and the patient cannot cooperate with treatment; (3) associated with other malignant tumors; (4) associated with severe cardiovascular and cerebrovascular diseases, metabolic disorders, and other diseases; (5) those who have contraindications to the drug in this study; (6) those who took palliative chemotherapy before inclusion in the study; (7) those who were complicated by severe abnormal coagulation function; or (8) pregnant or lactating women. This study was approved by medical ethics committee (approval no. 2019040557) of the above hospital.

### 2.2. Nursing Methods

①Environmental care: after admitted to the hospital, the patients were provided a good hospital environment, kept quiet and comfortable, kept the indoor air fresh, and the temperature and humidity were appropriate. The hospital should introduce the ward environment, reduce the unfamiliarity of patients, establish a harmonious relationship between nurses and patients, and improve patients' trust in nurses. ② Psychological care: because patients are prone to a large number of adverse reactions during chemotherapy, patients have many negative emotions psychologically, such as resistance, depression, anxiety, depression, and other emotional changes, which make patients prone to extremely uncooperative situations during treatment. Therefore, nurses should actively communicate with patients, by listening to patients' needs, correcting patients' misconceptions, imparting correct treatment information to patients, and creating a trusting nurse-patient relationship with each other. ③Dietary guidance [14]: nurses should analyze the nutritional status of patients, analyze the relationship between the nutritional status of the body and the recovery effect in detail, and formulate relevant dietary management manuals, provide targeted guidance combined with the contents of the manual, inform and record the type, eating time, and intake of the patient's three meals a day (inform the patient in detail about the staple food and salt intake), instruct the patient to eat more fresh fruits and vegetables, consume milk and meat products reasonably, drink plenty of water, pay attention to nutritional balance, and prohibit the consumption of sweets. ④Discharge guidance: for discharged patients, discharge guidance and follow-up should be done well, and the recent physical condition of the patients should be grasped by telephone and WeChat.

### 2.3. Treatment Methods

The single-drug group was treated with seggio (Guoyao Zhunzi H20100135, Jiangsu Hengrui Pharmaceutical Company, 20 mg*∗*42 S). The first dose of the drug should be adjusted reasonably following the body surface area. If the body surface area is less than 1.25 m2, 40 mg orally each time; 1.25–1.5 m2, 50 mg orally each time; and >1.5 m2, 60 mg orally each time, 2 times a day, after breakfast and after dinner, continuous medication for 14 d and drug withdrawal for 7 d. 21 d of medication was used as a medication cycle.

The joint group was treated with apatinib (Guoyao Zhunzhunzi H20140103, Jiangsu Hengrui Pharmaceutical Co., Ltd., 0.25 g*∗*10 tablets) on the basis of using siggio (see single-drug group for usage), 1 time/d and 250 mg/time. If the patient has no obvious response in the first cycle, it can be increased to 500 mg in the second cycle, and continuous taking for 21 d is one drug cycle. Both groups were treated for 6 cycles.

### 2.4. Observation Indicators

1. Evaluation of the patient's recent treatment effect: the standard is based on the objective treatment effect of solid tumors formulated by the World Health Organization [15], which is divided into 4 stages, namely complete remission (CR), stable disease (SD), partial remission (PR), disease progression (PD), and total response rate (RR). The patient can enter the second treatment cycle if it is judged that there is no disease pathological change or progression, RR = (CR + PR)  ÷ total number of cases × 100%.
2. Measurement of the quality of life: the quality of life was evaluated with the use of the Quality-of-Life Questionnaire-Core 30 (QLQ-30) developed by the European Institute of Oncology [16]. The QLQ-30 scale includes 1 quality-of-life evaluation scale, 5 functional evaluation scales, 30 single-scale items, and the item score is 0–100 points. The score is positively correlated with the quality of life.
3. Measurement of serum tumor marker levels in the two groups: 5 ml fasting venous blood was collected, and the blood samples were centrifuged (centrifugation speed 3 000 r/min and centrifugation time 15 min), and chemiluminescence was used to detect CA724 and AFP levels.
4. Measurement of inflammatory factors levels in the two groups: ELISA kits (Sigma, CA, USA) were used to detect IL-4 and IL-10 levels.
5. Measurement of the three-year cumulative survival rate: the two groups of patients were followed up by telephone and regular outpatient follow-up (once every 3 months), and each patient was followed up for at least 3 years.
6. Measurement of immune function in the two groups: alkaline phosphatase-anti-alkaline phosphatase-bridging enzyme staining method was used to determine T-cell subsets (CD4+/CD8+, CD8+, CD4+, and CD3+ levels).

### 2.5. Statistical Analysis

SPSS 22.0 statistical software (IBM, NY, USA) was used for data analysis. The *χ*^2^ test was used to measure enumeration data, and these data were expressed as cases (%). The *t*-test was used to analyze measurement data, and these data were expressed as the mean ± standard deviation (*x* ± *s*). *P* < 0.05 means the difference is statistically significant.

## 3. Results

### 3.1. Measurement of Clinical Efficacy in the Two Groups

The total effective rate of the single drug group was 55.10%, which was lower than that of the joint group (81.63%) after treatment, as shown in Table 1.

### 3.2. Measurement of the Levels of Inflammatory Factors

After treatment, IL-4 levels were obviously decreased in the two groups, and IL-4 levels in the joint group was reduced relative to single-drug group (Figure 1(a)). Moreover, IL-10 levels were obviously decreased in the two groups, and IL-10 levels in the joint group was decreased versus to the single-drug group (Figure 1(b)).

### 3.3. Measurement of the Quality-of-Life Scores

After treatment, the quality-of-life scores and total scores in both groups were markedly increased, when compared to before treatment, and the single-drug group's quality-of-life scores and total scores were increased obviously compared to the joint group, as shown in Table 2.

### 3.4. Measurement of the Immune Function

As shown in Figure 2, CD4+/CD8+, CD4+, and CD3+ levels were increased, while the CD8+ levels were decreased in the two groups, and the changes of each index in the joint group were more significant than those in the single-drug group after treatment.

### 3.5. Measurement of Tumor Marker Levels

After treatment, the serum CA724 level of the joint group was 30.72 ± 3.13, and the AFP level was 5.22 ± 1.44; the serum CA724 level of the single drug group after treatment was 39.76 ± 3.10, and the AFP level was 8.16 ± 1.43. There were statistically significant differences between the same group and between the two groups, as shown in Figure 3.

### 3.6. Measurement of Three-Year Cumulative Survival Rates

Comparison with the single-drug group (20.41%), the three-year cumulative survival rate in the joint group (44.90%) was elevated markedly, as shown in Figure 4.

### 3.7. The Relationship between Tumor Marker Expression and Survival Time in Joint Group

As shown in Figure 5, the median survival time of patients with high and low expression of CA724 in the joint group was 17.5 months and 29 months, respectively, and the median survival time of patients with high and low expression of AFP was 19 months and 31 months, respectively, and the difference was statistically significant.

## 4. Discussion

Gastric cancer is a malignant tumor with high incidence and high mortality in China. There are no obvious symptoms in the early stage. Most patients are in the late stages when they are diagnosed. They may experience symptoms such as weight loss, decreased appetite, epigastric discomfort, and dysphagia. Quality of life is seriously affected. Because of the long-term stress of mind and body, patients with gastric cancer often have anxiety and depression, which is not conducive to the treatment of the disease, and will lead to a decrease in the treatment effect of the disease. Studies have shown [17, 18] that comfortable nursing care for patients with gastric cancer can effectively alleviate the patients' unhealthy psychology, maintain the nutritional balance of patients, and achieve high-quality clinical effects.

The treatment options for patients with advanced gastric cancer are limited. The main goal of treatment is to control the primary or metastatic lesions, improve the symptoms of patients, improve the quality of life of patients, and prolong the survival period of patients. Chemotherapy stops tumor cells from spreading and improves patients' quality of life. Seggio [19] has definite curative effect and high safety for advanced gastric cancer, but the single-drug efficacy is limited. Both tumor proliferation and metastasis depend on angiogenesis, and apatinib is a small-molecule vascular endothelial growth factor receptor inhibitor that can target tumor angiogenesis, thereby reducing the inflammatory response of patients and improving the symptoms of patients, and the normal cytotoxicity is low and the safety is good [20].

CA724 is a relatively common type of nonspecific tumor marker, which has extremely high sensitivity for non-small cell lung cancer and gastric cancer, and its sensitivity for diagnosing gastric cancer is about 60% [21, 22]. AFP is a commonly used tumor serum marker, and its level is low in healthy adult serum, but its level is increased in hepatocellular carcinoma [23]. A study reported [24] that serum AFP levels in gastric cancer patients after surgery were significantly lower than those before surgery. This suggests that serum AFP can be used for prognosis evaluation of gastric cancer patients. This study discovered that the clinical efficacy in the joint group was better than single drug group, and the serum CA724 and AFP levels after treatment were lower than those in the single drug group. The reason for the analysis is that the combination of apatinib and seggio can play a synergistic effect, selectively inhibit tumor angiogenesis, induce tumor cell apoptosis, and reduce serum tumor marker levels. This study also displayed that IL-4 and IL-10 levels in the joint group were decreased obviously relative to the single-drug group; the CD4+/CD8+, CD4+, and CD3+ levels in the joint group were remarkably elevated, while CD8+ levels were obviously decreased compared to the single-drug group; and the three-year survival rate in the joint group was remarkably upregulated compared to the single-drug group. After treatment, the quality-of-life scores and total scores of the joint group were markedly elevated relative to the single-drug group. These data indicated that the combination of apatinib and seggio can reduce the inflammatory response, enhance the immune function, and improve the quality of life and survival time of patients. Under normal circumstances, the two are in a state of balance. If the balance is broken, it is easy to cause diseases. In gastric cancer patients, the ratio of Th1/Th2 cytokines is unbalanced, and IL-10 and IL-4 levels are significantly increased, which leads to the immune suppression of the body and the continuous proliferation of tumor cells [25]. Apatinib can selectively suppress the proliferation of tumor cells, regulate the balance of Th1/Th2 cytokines, and then reduce IL-10 and IL-4 levels.

## 5. Conclusions

Apatinib combined with seggio has a high clinical effect on patients with advanced gastric cancer undergoing comfort nursing intervention. The pain of the patient's treatment is better than that of seggio alone.

## Figures and Tables

**Figure 1:** Measurement of inflammatory factors levels.  ^*∗*^*P* < 0.01 vs before treatment, ^#^*P* < 0.01 vs joint group. (a) Detection of IL-4 levels in the two groups; (b) Detection of IL-10 levels in the two groups.

**Figure 2:** Measurement of immune function. *∗P* < 0.01 vs before treatment. #*P* < 0.01 vs joint group. (a) Measurement of CD3+ levels in the two groups. (b) Measurement of CD4+ levels in the two groups. (c) Measurement of CD8+ levels in the two groups. (d) Measurement of CD4+/CD8+ levels in the two groups.

**Figure 3:** Measurement of tumor marker levels in the two groups. (a) Measurement of CA724 levels. (b) Measurement of AFP levels.

**Figure 4:** Measurement of three-year cumulative survival rates.

**Figure 5:** The relationship between the expression of tumor markers in the joint group and survival time. (a) The relationship between CA724 expression and survival time. (b) The relationship between AFP expression and survival time.

**Table 1:** Measurement of clinical efficacy (*n*, %).

Group	*n*	CR	PR	SD	PD	Total effective rate
Joint group	49	23	17	7	2	40 (81.63)
Single-drug group	49	14	13	13	9	27 (55.10)
X^2^						8.977
*P*						0.030

**Table 2:** Measurement of quality-of-life scores (*x* ± *s*).

Group	n	Physical function		Emotional function		Cognitive function		Social function		Role function		Total score	
		Before treatment	After treatment	Before treatment	After treatment	Before treatment	After treatment	Before treatment	After treatment	Before treatment	After treatment	Before treatment	After treatment
Joint group	49	53.22 ± 4.90	82.69 ± 4.66*∗*^△^	53.20 ± 4.99	83.04 ± 5.01*∗*^△^	56.29 ± 4.56	84.37 ± 4.76*∗*^△^	54.29 ± 4.82	85.04 ± 4.46*∗*^△^	53.29 ± 5.32	82.86 ± 5.55*∗*^△^	54.18 ± 4.89	82.88 ± 5.35*∗*^△^
Single-drug group	49	54.27 ± 4.70	67.41 ± 4.88*∗*	53.90 ± 4.48	67.47 ± 4.70*∗*	57.47 ± 4.62	71.45 ± 4.83*∗*	55.12 ± 4.65	69.18 ± 4.17*∗*	54.31 ± 4.54	67.88 ± 4.99*∗*	54.71 ± 4.35	68.00 ± 4.56*∗*
t		1.073	15.86	0.724	15.87	1.277	13.34	0.875	18.18	1.021	14.06	0.568	14.82
*P*		0.286	≤0.001	0.471	≤0.001	0.205	≤0.001	0.384	≤0.001	0.310	≤0.001	0.571	≤0.001

*∗P* < 0.01 vs before treatment, ^△^*P* < 0.01 vs joint group.

## Data Availability

Data to support the findings of this study are available on reasonable request from the corresponding author.
